The article "Construction of Rural Tourism Brand Value Management Model from the Perspective of Big Data" was published in 2022. Journal: Comput Intell Neurosci.

# Construction of Rural Tourism Brand Value Management Model from the Perspective of Big Data

**DOI:** 10.1155/2022/5623782

**Published:** 2022-07-22

**Authors:** Wenlong Wang, Daihanyu Wu

**Affiliations:** ^1^School of International Education, Guizhou Normal University, Guiyang 550001, Guizhou, China; ^2^School of Computer Science, Nanjing University of Posts and Telecommunications, Nanjing 210046, Jiangsu, China

## Abstract

Rural tourism has become an important branch of tourism management. Big data technology provides tools for rural tourism brand value management. This study aims to build a brand value management model for rural tourism from the perspective of big data. The rural tourism brand value management model under the big data perspective takes the rural tourism brand competitiveness as the starting point to analyze the relationship between brand value and brand competitiveness, so that the brand competitiveness under the perspective of rural tourism brand value has a more specific and quantifiable index system. From the two aspects of enterprise value advantage and customer value advantage, this article looks for the factors that comprehensively reflect the brand competitiveness of rural tourism. After the establishment of the index system, the BP neural network model is used to make the multiple factor evaluation more objective and feasible. Finally, it is proposed to enhance the competitiveness of rural tourism brands from the perspective of the reconstruction of competitive advantage based on enterprise value and the reconstruction of competitive advantage based on customers.

## 1. Introduction

The rapid development of rural tourism has played a positive role in the economy and life of rural areas [1–3]. Since rural tourism has played an important role in promoting economic development and improving living standards in rural areas, vigorously developing the rural tourism industry has gradually become one of the industries promoted by the government [4–6]. However, the problems faced by rural tourism also follow [7–12]. For example, some rural tourism brands have a single supply structure, resulting in a mismatch between supply and demand. The simplification and homogeneity of rural tourism products have also seriously hindered the driving effect of rural tourism on the economic development of rural areas These problems reduce tourists' willingness to visit and revisit rural tourism destinations, and seriously hinder the sustainable development of rural tourism enterprises.

Today, with the homogenization of products, the brand-based business model has become the main form that dominates the fate of the company [13]. If the brand is correctly used, it can become sustainable and effective competitiveness that creates unlimited value. A strong brand can obtain a significant premium effect [14–20]. The core value of the brand is unique and occupies a unique position in the hearts of customers. The brand trademark is protected by law and has a leading position. The brand can integrate the internal and external resources of the enterprise. The brand has the ability to extend into other markets and industries. The brand trademark is unique to the enterprise [18]. The strong brand value is regarded as the representative of the enterprise with a huge market share and will not be sold. Therefore, brand competitiveness not only includes the comprehensive advantages of enterprises in resources, capabilities, technology, management, marketing, human resources, and so on but also has strong practicality and operability.

Big data technology [21–24] has been booming in recent years, and has affected all aspects of social life, including rural tourism. Therefore, it is necessary to conduct an in-depth discussion and investigation on the brand value management of rural tourism from the perspective of big data, so as to find new solutions for the homogenization and simplification of rural tourism products.

## 2. Overall Research Framework

In the rural tourism industry, brand competitiveness evaluation is an important part of brand value evaluation. The evaluation method of brand competitiveness based on brand value in this article is closely related to the evaluation method of brand value. The representative methods for evaluating brand value from the perspective of enterprises include the interbrand evaluation method and the “MSD” evaluation method [16–19]. The idea of the interbrand evaluation method is that the brand value is equal to the product of the brand revenue and the brand multiplier.

Brand strength can be converted into brand multipliers. However, there are still some shortcomings in this method. For example, the future sales forecast in this method is based on the present. Due to the fierce market competition and changing circumstances, the brand's past sales situation may not be able to continue in the market. Second, it is difficult to determine the rate at which the brand is separated from intangible assets to form income. Furthermore, this method does not consider the influence of consumers on brand value. The MSD method defines three indicators that reflect the competition of Chinese brands and the status of Chinese brand value, namely, the brand's market shareability (*M*), the brand's excess profit-making capacity (*S*), the brand's development potential (*D*), and the brand value. It is equal to the sum of the products of the three scores multiplied by the corresponding weights. This evaluation method is currently the largest system in the relevant research field in China. Still, the limitation of this method is that the idea of taking market share as the core does not have long-term advantages; it does not distinguish the difference between company value and product brand value and can only evaluate generic brands. Finally, it also does not consider the factors of consumers.

Consumer-based brand value evaluation methods are primarily based on the relationship between the brand and consumers and obtain a qualitative evaluation of brand value through consumer surveys. The brand evaluation models proposed by foreign scholars mainly include the Brand Equity Ten model and the consumer-based brand value model, which are qualitative evaluations. The Loyalty Factor Rule is an attempt by domestic scholars to evaluate the brand value based on consumers quantitatively [20]. These models fully affirm the important role of consumers in brand value, but they also have some limitations. First, the influence of the enterprise on the brand value is not considered. Second, these models are not easy to quantify. They use some statistical tools to analyze the brand's value through surveys and interviews with consumers, so it is tough to convert the relationship between consumers into the value of the brand value, which limits its scope of application to a certain extent.

The brand value evaluation method based on the enterprise evaluates the value of the brand through the enterprise's financial status and the brand's market performance. Most of them are quantitative methods, but they do not consider the influence of consumers on the brand value; the brand value evaluation method, based on the consumer's point of view, considers the brand's value from the perspective of consumer relations. Most of them are qualitative methods, which are difficult to give exact credibility, and they also ignore the influence of the enterprise on the brand value. Therefore, this article attempts to evaluate brand competitiveness from the comprehensive perspective of brand enterprise value advantage and customer value advantage; trying to build quantitative and comparable indicators of consumer value and brand-consumer equity assets that are difficult to quantify. It is a pioneering innovation in evaluating brand competitiveness to avoid the distribution of weights among factors as much as possible.

Based on the above analysis, the rural tourism brand value management model under the big data perspective built in this study is shown in Figure 1, which presents the technical route of this study.

## 3. Application Principles of Evaluation Method for Rural Tourism Brand Competitiveness

Before designing the measurement standards and measurement indicators of rural tourism brand competitiveness, a set of corresponding principles should be established to prevent the design of indicators from deviating from reality. Indicator design should follow the following principles:

The first is the principle of representation. Many indicators affect rural tourism brand competitiveness, but not all aspects can be put into the evaluation indicator system. Representation requires that the design of evaluation indicators reflect the primary objective manifestation of various factors of rural tourism brand competitiveness.

The second is the system principle. Each object of evaluation can be called a self-contained system. Therefore, the new method should be constructed according to the system's thinking, using the relationship between the method system and the outside and the relationship between the indicators in the system to form an open and interactive method system.

The third is the principle of effectiveness. Effectiveness means that the evaluation indicators of brand competitiveness should be clear, simple, and intuitive. The number of indicators is appropriate. There is no overlap and repetition between indicators, but try to reflect the general or common characteristics of the evaluation object to improve the feasibility and comparability of the actual evaluation.

The fourth is the principle of practicality. The purpose of designing rural tourism brand competitiveness evaluation indicators from the perspective of rural tourism brand value is to measure the strength of corporate brand competitiveness, which should reflect the practical significance of evaluation indicators. That is to say, the evaluation indicators should become a powerful tool for enterprises to self-diagnose and improve themselves and continuously improve the weak points of enterprise brand building to establish a competitive brand finally.

## 4. Rural Tourism Brand Competitiveness Evaluation Index System from the Perspective of Brand Value

This article will establish the evaluation index system of rural tourism brand competitiveness from the brand's enterprise value advantage and the brand's customer value advantage.

### 4.1. Rural Tourism Brand's Enterprise Value Advantage Index

The brand's entrepreneurial advantage reflects the rights and interests that the brand brings to the enterprise in the competition. This article mainly reflects the asset value and equity value of the brand and mainly draws on the factors of the Interbrand law and the MSD law to describe.

#### 4.1.1. Rural Tourism Brand Asset Value Advantage Index

The asset value advantage of the brand mainly refers to the value of the brand as an intangible asset, which is reflected in the market position advantage of the brand, the internal support advantage of the enterprise, and the brand development advantage. Each factor is explained in detail:

(1) Market position advantage: market shareability, overvalue profitability, market stability, and the brand's position advantage. It should not only reflect the current market position but also reflect that the brand's profitability is continuous and stable. This article selects quantitative and external indicators directly related to brand market competitiveness. The market position is mainly reflected in market shareability, value-added profitability, and market stability indicators. The market shareability reflects the current market share of a brand relative to similar competitors, which can be obtained by analyzing the company's market share, market sales, and turnover rate of total brand assets. The profit advantage of the brand relative to its competitors reflected by the super-value profitability is reflected in the brand premium, the rate of return on brand equity, and the sales profit rate. Market stability is reflected in the consistency and consistency of the brand in the sales market of a specific customer group, reflected in the growth rate of sales revenue, the number of consecutive profitable years, and the age of the brand. These specific indicator values can be obtained from within the enterprise. The specific performance factors of the above indicators are calculated as follows:
  (1) $$\begin{array}{c} \text{Market share}=\text{market share of the brand,}\\ \text{Market sales}=\text{sales of brand products}\times \text{unit price of brand products,}\\ \text{The turnover rate of total brand assets}=\frac{\text{net brand sales revenue}}{\text{average total assets}}\times 100\%,\\ \text{Brand premium}=\text{branded product price}-\text{unbranded product price,}\\ \text{Return on assets}=\frac{\text{brand profit}}{\text{total enterprise assets}}\times 100\%,\\ \text{Brand sales profit margin}=\frac{\left(\text{brand product sales}-\text{brand product cost}\right)}{\text{sales}},\\ \text{Sales revenue growth rate}=\frac{\left(\text{sales revenue of original brand products}-\text{sales revenue of brand products in the previous year}\right)}{\text{sales revenue of brand products in the last year}}. \end{array}$$
The number of consecutive profitable years and brand age can be obtained from direct data.
(2) Internal support advantages of the enterprise: brand quality support, brand technology innovation, brand resource financing and supply, and brand marketing ability.
The indicators mentioned above of an enterprise's internal support advantages complement each other, promote each other, and guarantee each other. Together, they form a solid foundation for brand competitiveness and are also the fundamental reason brands can create value advantages.
  (a) Brand quality support: brand quality not only has internal functional quality requirements but also pays attention to external quality and extension quality (service quality); brand quality includes not only the quality of the brand itself but also the quality embodied by the brand, that is, the quality of the brand in the minds of consumers. While improving product quality, we must prioritize improving the quality of consumers' psychological feelings so that that product quality can be transformed into quality recognized by customers. The specific manifestations of common brand quality support are pass rate, rejection rate, level product output value growth rate, etc.
  (b) Brand technological innovation: brand technology innovation refers to the improvement of brand design, materials, processes, devices, etc., or the creation of new products by enterprises using relevant knowledge and experience. Effective technological innovation is conducive to reducing the uncertainty of the brand's future, giving the brand greater market control power in the competitive environment, and improving the brand's competitive advantage. Accelerating technological innovation first requires increasing capital investment. Throughout the process of the emergence and development of strong brands in the world, it is inseparable from increasing investment in scientific and technological research and development. Second, it is necessary to change the orientation of technological innovation. Technological innovation is not a purely technical issue but technological innovation in a market environment. Enterprises must build technological innovation based on market orientation and emphasize the customer orientation of technology. Therefore, in the organizational structure of technological innovation, it is necessary to change from the original “serialized technological innovation” organization to a team-oriented “simultaneous technological innovation” organization. The brand's technological innovation is embodied in the replacement rate of new products, the speed of new product development, the coefficient of investment in technological innovation, and the proportion of technical expenditures in sales revenue.
  (c) Brand resource financing ability: the operation of any brand is inseparable from the support of resources. The financing and supply of resources are embodied in the financing and supply of people, money, and materials. Funding for a competitive brand can be obtained from two sources: first, relying on the market influence of strong brands to increase sales volume and unit profit level and enhance the ability to raise funds through self-accumulation; second is to rely on the brand's value-added ability and social influence and fully use the brand's market appeal. To promote social capital to gather in strong brand enterprises, the brand's ability to raise funds can be measured from the aspects of the enterprise's credit rating, debt level, and the state's support for the industry. The raw material energy supply capacity can be assessed by the unit raw material energy cost, the number of suppliers with special cooperative relations, and their status in the industry. People are the most important and dynamic resource among various resources of an enterprise. The quantity and quality of supply of people directly determine the competitive advantage of an enterprise. The ability to raise human resources can be measured by the enterprise's shortage of various human resources.
  (d) Brand marketing power: the evaluation of brand marketing power can be considered from three perspectives: marketing innovation, marketing execution, and marketing management capabilities. The degree of marketing innovation is mainly evaluated from the perspective of whether an enterprise continuously invests and combines marketing resources and launches creative marketing plans to meet customer needs and guide customer needs. Marketing execution mainly considers whether the enterprise can execute the formulated marketing plan and make control efforts according to the changing market environment. Marketing management capabilities are mainly evaluated by maintaining and developing relationships with suppliers, distribution channels, the public, and customers.
(3) Brand development advantages: brand strategic investment, growth index, and acceptance of extending new products. The brand's asset value is reflected in the market advantage it can bring to the enterprise in the current period and the development potential and expansion ability, which is reflected in the brand extension and potential value of expansion. Brand extension and expansion can extend contributions from existing brand equity to new products, including brand name, consumer attitudes toward the brand, adaptability between existing and extended products, consistency of brand image, etc. Therefore, it is mainly reflected in the company's strategic investment in the brand, the brand growth index, the acceptance of extended new products, and the replacement rate of new products. These performance factors are specific and quantifiable data, and the specific calculation methods are as follows:
  (2) $$\begin{array}{c} \text{Brand strategic investment}=\frac{\left(\text{expected brand investment}-\text{current brand investment}\right)}{\text{current brand investment}},\\ \text{Growth index}=\frac{\left(\text{market share of a brand in this year}-\text{market share of the brand in the previous year}\right)}{\text{market share of the brand in the last year}}\times 100\%,\\ \text{Extended new product acceptance}=\frac{\text{current new product sales}}{\text{new product production}}. \end{array}$$

#### 4.1.2. Rural Tourism Brand Equity Value Advantage Index

The equity value advantage of a brand is a theoretical framework system for evaluating and managing brand value purely from the perspective of the relationship between consumers and brands. The indicators mainly reflect the mental resources of consumers owned by enterprises. This article integrates Keller's CEBA model and Aaker's ten-factor brand model and considers the customer's brand equity value advantage from the following aspects:

*(1) Brand Awareness*. Awareness without prompting, awareness after prompting, and subjective familiarity with the brand. Brand awareness refers to how consumers can remember or know a certain brand when they mention a certain type of product. Brand awareness plays a vital role in consumers' purchase or consumption decisions. The higher the brand awareness, the easier the brand is to be accepted by consumers when purchasing or consuming; Due to the constraints of time, energy, knowledge, and experience in judging product quality, consumers often decide to buy or consume the brands they think are the most well-known and familiar. Brand awareness can be measured in many ways. This article measures it through three indicators: unprompted first awareness, post-prompt awareness, and consumers' subjective familiarity with the brand. The brand's unprompted first awareness refers to the consumer who, without any prompting, the percentage of people who first thought of the brand as a percentage of the total surveyed. Its calculation formula is as follows:

(3) $$\begin{array}{c} \text{Awareness without prompting first popularity}=\frac{\text{number of people who answered the brand name first}}{\text{number of respondents}}. \end{array}$$

Awareness after prompting refers to the percentage of people who can think of the brand when consumers are prompted to the total number of people surveyed. Its calculation formula is as follows:

(4) $$\begin{array}{c} \text{Subjective familiarity with the brand}=\frac{\text{the number of people who answered the brand name after the prompt}}{\text{the number of respondents}}. \end{array}$$

The subjective familiarity of a brand refers to the subjective measurement description of consumers' familiarity with a certain brand. It can be distinguished by setting scores and other comparative measurement methods, allowing consumers to rate the familiarity of different brands; the higher the score, the more subjectively familiar consumers are with the brand.

Obviously, the higher the measurement value of the above three indicators, the higher the brand awareness.

*(2) Brand Associations*. Functional associations, organizational associations, and brand uniqueness. Brand association refers to the depth and breadth of things consumers can associate with a brand name, including the appearance of brand products, the quality of products and services, functional benefits, corporate image, product characteristics, brand personality and symbols, and other associations of customers. Brand associations help consumers process and extract information, differentiate brands, generate reasons for purchase, and influence consumer attitudes. Brand association is formed by long-term contact between customers and brands. Consumers have different associations with different brands to reveal the differences between brands. This article analyzes consumers' associations with brand functions, organization associations, and brand uniqueness from several aspects.

The functional association and organizational association of a brand mostly reflect the strength of the brand association. The uniqueness of a brand refers to consumers' ability to feel that it can provide a different value for themselves compared with other similar brands. This article will measure brand uniqueness from customers' subjective and holistic perspectives without further disaggregating it into the product, service, emotional function uniqueness, etc.

The above three indicators are all assessed through the customer evaluation scale. The higher the evaluation, the stronger the brand association.

*(3) Brand Recognition*. Brand symbol recognition, brand image recognition.

Brand symbols are also an effective condition for customers to recognize and purchase brand products. It is an external and specific thing of the brand, which can directly give consumers a strong visual impact. Brand symbols mainly include brand name, logo, packaging, color, etc. Brand awareness in this article refers to the consumer's awareness and understanding of brand symbols. Generally speaking, the higher the consumers' awareness of a brand, the stronger their ability to recognize and recall the aspects mentioned above related to the brand and vice versa. Brand image mainly refers to the corporate image, which generally refers to the customer's intuition and feeling about the company's philosophy and the quality of employees in the process of obtaining products.

This article adopts the method of measuring consumers' awareness of brand symbols and brand image to quantify and deal with them and consider them in the form of a seven-level scale. The higher the customer response value, the better the brand recognition.

*(4) Customer Loyalty*. Brand price loyalty, behavior loyalty, and customer trust.

Different scholars have classified brand loyalty in many ways, one of which is to classify it into emotional and behavioral loyalty. Emotional loyalty means that the brand personality is consistent with consumers' lifestyles, values, etc., so consumers will have certain feelings for the brand and then reach the brand's level of familiarity and promotion. Behavioral loyalty refers to the behavior of consumers continuing to buy a brand. The measurement methods of brand loyalty can be roughly divided into four categories: measurement by purchase ratio, measurement by continuity of purchase behavior, the measure by the length of time that a brand is the main purchase or consumption brand, and measurement by attitude toward the brand, this article reflects on three aspects of measurement methods: price loyalty, behavioral loyalty, and trust.

Price loyalty is the most direct response to brand loyalty; when the price of the brand increases or the price of similar competitors decreases, the possibility of consumers still insisting on buying branded products, which is the most direct equity value to the enterprise generated by behavioral loyalty, which can be measured by the price increase loyalty index and the price decrease loyalty index.

Behavioral loyalty is also reflected in the repeated consumption of customers. The number of people who still buy the brand within two purchase cycles is reflected in the repeat purchase rate. Brand trust refers to the overall degree of trust consumers have in a brand, which is objectively expressed as the unsuspecting psychological reaction of consumers in the process of using the brand.

Brand trust can be decomposed into many sub-indices for measurement. Still, this article mainly reflects it from an overall perspective, expressed as the customer recommendation rate, the proportion of consumers who recommend the brand's products to others in a period to the total number of purchasers.

Among the above indicators, the specific indicators that can be measured are as follows:

(5) $$\begin{array}{c} \text{Price increase loyalty index}=\frac{\text{brand price increase rate of change}}{\text{market share rate of change}},\\ \text{Markdown loyalty index}=\frac{\text{Rate of Change in Major Competitors' Markdown}}{\text{Rate of Change in Market Share}},\\ \text{Repeat purchase rate}=\frac{\text{the number of people who repeatedly purchased the brand's products during the period}}{\text{the total number of purchasers of the brand during the period}},\\ \text{Customer referral rate}=\frac{\text{the number of people who recommend the brand to others}}{\text{the total number of purchasers of the brand}}. \end{array}$$

### 4.2. Rural Tourism Brand's Customer Value Advantage Index

The customer value advantage of a brand is the utility evaluation of the transfer value of the brand by customers in the dynamic consumption process, which can be divided into functional value advantage, emotional value advantage, and monetary value evaluation advantage.

(1) Functional value advantage: the functional value of a brand refers to the customer's subjective perception of the physical value of a brand. The customer's value judgment of a certain brand belongs to an external cognitive orientation. The functional perceived value of a brand has the following salient features: the first is subjectivity; that is, the perceived value is determined by the customer's subjective judgment, which may be inconsistent with the brand's perception of the brand's product or service value; the second is multi-dimensionality, which includes functional value and nonfunctional value, and is a perception generated by customers in the process of consumption or use; the third is a hierarchy; that is, functional value and various nonfunctional value form a ladder from low to high. Generally, only after the low-level value is satisfied the high-level value will appear; the fourth is comparability, which is not only the result of the customer's comparison of perceived income and perceived effort but also the result of the comparison of competing enterprises; the fifth is contingency. Different consumers have different perceptions of the same brand, even if the same customer has different perceptions of the same brand in different consumption environments.
This article considers the measurement of brand functional value advantage from an overall perspective. The functional value advantage of the brand reflects the satisfaction function of product attributes, product performance satisfaction function, product quality satisfaction function, and product safety satisfaction function. For the specific evaluation of these indicators, this article takes the form of a customer questionnaire to allow customers to score these aspects of the brand product. The higher the score, the higher the functional value advantage.
(2) Emotional value advantage: it mainly reflects the noneconomic emotional value given to customers in the process of brand consumption. It can reflect the brand's emotional value advantage from three aspects: experiential benefits, symbolic benefits, and satisfaction of consumers' psychological needs.
  - Experiential benefits: consumers' subjective feelings about the shopping environment and personnel in the process of purchasing products or enjoying services. Such benefits mainly meet subjective requirements. It is primarily reflected in the satisfaction of the shopping environment and the recognition of the service level of the waiters.
  - Symbolic benefits: the additional benefits of consuming a product or service are an external advantage, usually reflecting non-product-related attributes. Mainly to satisfy implicit needs such as social identity, personal performance, and personal self-esteem. Consumers care about the status, exclusivity, and fashion of a brand because it reflects the consumer's self-positioning and image.
  - Satisfaction of consumers' psychological needs: the emotional utility of the brand's consumption can be reflected in comparing consumers' psychological expectations and actual purchases.
The specific indicators of the above three criteria layers are all based on customer perception and are qualitative indicators without specific quantitative indicator values. In this article, the service and feelings provided by customers to the brand are obtained by designing a questionnaire and quantified according to the customer evaluation level.
(3) Monetary value evaluation advantage: this indicator mainly measures the customer value advantage of the brand from the customer's perceived price benefit because the most direct and obvious payment of customer consumption is currency. Of course, the brand must be expressed as a high price for similar products, so consumers, when choosing brand products, try to pursue that the expected purchase cost is greater than the perceived purchase cost. Otherwise, consumers may switch to other brands. The expected purchase cost refers to the price that consumers make in the mind of the brand product before purchasing, and the brand with its perfect quality and service, the customer perceives that the purchase price seems to be much lower, that is, the perceived price benefit is large so that the brand can be attractive and competitive.

This article quantifies the perceived price benefit through the questionnaire's consumer evaluation level. The higher the evaluation value, the higher the monetary value evaluation advantage.

Based on the above analysis, the overall index system of brand competitiveness is summarized as shown in Table 1.

## 5. Application of BP Neural Network Method in Rural Tourism Brand Competitiveness Evaluation

At present, the methods adopted by many scholars to evaluate brand competitiveness mainly include the analytic hierarchy process, multiple regression analysis methods, fuzzy comprehensive evaluation method, etc. These methods have their insurmountable shortcomings [25–29]. In recent years, the emergence of neural networks has provided new ideas for multi-index systematic evaluation. Neural networks have many excellent characteristics, are best at making decisions on approximate, uncertain, and even contradictory knowledge environments, and can solve artificial weight design and calculation of correlation coefficient.

### 5.1. The Basic Principle of Artificial Neural Network

The BP neural network [25–29] is developed based on the back-propagation algorithm. It is a multi-level feedback network with error back-propagation. It uses the tutor learning algorithm and consists of input, hidden, and output layer nodes. There is no association between nodes at the same layer and forward connections between nodes at different layers. Its algorithm idea is to take a pair of learning modes, process the input mode through the network input layer, hidden layer, and output layer by layer to obtain an output mode, and calculate the error between the network output mode and the expected output mode. The error is transmitted in the reverse order of the output, hidden, and input layers. The connection weight of each layer is corrected layer by layer in the direction of reducing the error. Repeat the above process until the output error of each pair of learning modes and network meets the requirements.

### 5.2. Rural Tourism Brand Competitiveness Evaluation Model Based on BP Neural Network

#### 5.2.1. Determination of Artificial Neural Network Model Structure

Generally speaking, a three-layer BP network is used: input layer, hidden layer, and output layer. The number of nodes in the input and output layers can be directly selected according to the specific research object. For the problem of determining the relationship between multiple variables, the independent variable is usually the input item, and its number is the number of nodes in the input layer; the dependent variable is the output item and the number of nodes in the output layer is 1. The number of hidden layer nodes reflects a certain extent, the ability of the network to learn the degree of correlation between the input vector and the output vector from the training samples, so if the number of hidden layer neurons is too large, it is easy to slow down the network calculation convergence speed, even the network is in an infinite loop and cannot converge; if the number is too small, the intrinsic relationship between the input vector and the output vector in the training sample may not be fully learned. This will affect the training and prediction accuracy of the network, which is imperfect for the network itself. In the brand competitiveness model, the target layer is brand competitiveness A, the criterion layer is B1–B10, the factor layer includes indicators C1–C29, and the 29 indicators of the factor layer are taken as the input layer, respectively *X* (C1)–*X* (C29), then the number of nodes in the training layer is 59 (according to experience: for a neural network with *m* input nodes, (2*m* + 1) hidden nodes will achieve good results between network capacity and training time), and the output layer is the target layer.

#### 5.2.2. Determination of the Input Layer

There are qualitative and quantitative indicators among the 29 indicators involved in the evaluation index system. According to the evaluation criteria of the indicators, the indicators are divided into positive indicators and reverse indicators. Since different indicators reflect brand competitiveness from different perspectives, there is no direct comparison between indicators. To facilitate the determination of the final evaluation value and consider the convergence problem of neural network training, it is necessary to perform dimensionless processing on the indicators. The first is the standardization and normalization of the evaluation indicators. That is to say, a method of eliminating the influence of indicators and dimensions through certain mathematical transformations and converting indicators with different properties and dimensions into a quantitative value that can be comprehensively evaluated.

Positive indicators are generally described by the following linearly increasing function:

(6) $$\begin{array}{c} y_{i}=\left\{\begin{array}{cc} 0 & x\left(c_{i}\right)\leq x_{\text{min}}\left(c\right),\\ \frac{x\left(c_{i}\right)-x_{\text{min}}\left(c\right)+0.01}{x_{\text{max}}\left(c\right)-x_{\text{min}}\left(c\right)+0.01} & X_{\text{min}}\left(c\right)\leq x\left(c_{i}\right)\leq x_{\text{max}}\left(c\right),\\ 1 & x\left(c_{i}\right)\geq x_{\text{max}}\left(c\right). \end{array}\right. \end{array}$$

The inverse indicator uses the following dimensionless standard function:

(7) $$\begin{array}{c} y_{i}=\left\{\begin{array}{cc} 0, & x\left(c_{i}\right)\leq x_{\text{min}}\left(c\right),\\ \frac{x_{\text{max}}\left(c\right)-x\left(c_{i}\right)+0.01}{x_{\text{max}}\left(c\right)-x_{\text{min}}\left(c\right)+0.01}, & x_{\text{min}}\left(c\right)\leq x\left(c_{i}\right)\leq x_{\text{max}}\left(c\right),\\ 1, & x\left(c_{i}\right)\geq x_{\text{max}}\left(c\right). \end{array}\right. \end{array}$$

The hidden layer of the network selects the Sigmoid function as the excitation function, that is:

(8) $$\begin{array}{c} f\left(x\right)=\frac{1}{1-e^{-x}}. \end{array}$$

#### 5.2.3. Selection and Improvement of Network Algorithms

The learning algorithm of the BP neural network is based on gradient descent, which is easy to make the solution of the problem fall into the local minimum. Momentum factors, variable learning rates, etc., can be introduced to improve the convergence speed of the algorithm. In addition, combining the genetic algorithm and the neural network and using the genetic algorithm to assist the artificial neural network in training and optimizing the network weights can improve the algorithm's overall convergence speed and accuracy.

#### 5.2.4. Training Termination Test

The neural network has an optimal training number when the hidden layer nodes are determined. Generally, the test set method and the cross-validation method are used to judge the prediction error. When the prediction error is the smallest, the training is stopped. In the evaluation model of brand competitiveness, the index values of a part of the training samples are first entered into the network through the input layer. A part of the sample data is reserved as a test sample and does not participate in the training. The BP neural network compares the input value and the desired output value, then adjusts the connection weights of each layer of the neural network and the threshold of each neuron according to the function of the difference between the two, and finally minimizes the error function. During training, stop after a certain number of training sessions. Use the reserved test samples to test the test error of the network to the sample at this time. When it is found that the test error begins to rise, over-training may occur, but in general, the training continues, and the network is constantly tested with test samples; after many comparisons, the optimal number of training sessions is finally determined.

#### 5.2.5. Sample Selection and Organization

The selection of samples follows the following principles: enough samples, representative samples, and uniform distribution of samples. The test samples are randomly selected in many practical applications, generally 10% to 15% of the training sample capacity. In the brand competitiveness evaluation model, the actual operating data of some developed brands or other available brand products can be selected as training samples to train the neural network.

When the index value of the target brand is input into the neural network, the trained BP neural network can evaluate the rural tourism brand competitiveness of the product relatively objectively. The output value of the output layer is the judgment value of the rural tourism brand competitiveness. Through the judgment value, we can know the strength of the rural tourism brand competitiveness. The entire process is shown in Figure 2.

## 6. Case Analyzing

To test the feasibility of the model, this article selects the brand competitiveness of several rural tourism brands as the research object, which are denoted by *A*, *B*, *C*, *D*, *E*, *F*, *G*, *H*, and *I*. Each brand has its business characteristics.

According to the evaluation index system of rural tourism brand competitiveness, for the brand's asset value index, the quantifiable index data can be obtained from the data released by the corporate websites of various brands; for unmeasurable indicators, the author asked the professional personnel to give the data after professional evaluation. According to the index system, the author designed corresponding questionnaires for the brand equity value index and customer value advantage index. The data obtained from various channels need to be sorted and processed before being used as analysis data.

For the competitiveness of these rural tourism brands, we obtained relevant information through the brand evaluation network. The final ranking of rural tourism brands is *B*, *G*, *H*, and *I* (the four brands above are the most competitive brands), *A*, *C*, and *E* (the middle three brands are moderately competitive), *D* and *F* (these two brands are weakly competitive), and finally simulated the learning sample data of nine brands, as shown in Table 2.

Taking the data in Table 2 as the neural network's training sample, after the neural network's learning and training, the sum of squares of the network error reaches the error target of 10^−3^. The training process is shown in Figure 3.

The output value of the trained neural network is very close to the expected value, indicating that the model can accurately determine the competitiveness of rural tourism brands according to various evaluation indicators. Therefore, after the network model training is completed, the brand competitiveness model based on BP neural network has been established. When evaluating the competitiveness of other rural tourism brands, it is only necessary to input the index data after dimensionless processing of the evaluation samples. Then the evaluation results can be obtained.

A new rural tourism brand *J* has just entered the market. To determine the competitiveness of the brand, after dimensionless processing of the brand's index data, input the model to get

(9) $$\begin{array}{c} P\_\text{test}=\left[\begin{array}{c} 0.1123\;0.1814\;0.1778\;0.5734\;0.1923\;0.4544\;0.2309\;0.3156\\ 0.1912\;0.1045\;0.1857\;0.1917\;0.2125\;0.2027\;0.2536\;0.2147\;0.5067\;0.5608\\ 0.4001\;0.4222\;0.2031\;0.2461\;0.5672\;0.3223\;0.6445\;0.6823\;0.5677\;0.4509\;0.6801\prime \end{array}\right],\\ Y=\text{sim}\left(\text{net},P\_\text{test}\right)=\left[0.0001,0.0006,0.9998\right]. \end{array}$$

It means that the output of the trained network is very close to 001. That is to say, the brand's competitiveness is determined to be weak. It can prove the feasibility and effectiveness of the model. Enterprises should diagnose the problem of rural tourism brand management, choose the correct investment direction, and enhance the rural tourism brand's competitiveness.

## 7. Conclusions

Based on the theoretical research on rural tourism brand value management by domestic and foreign scholars and the investigation of corporate brand management practices, this article establishes a rural tourism brand value management model from the perspective of big data. Through the evaluation of rural tourism brand competitiveness, this article puts forward methods and countermeasures to improve brand competitiveness based on value advantage reengineering. This study defines the brand competitiveness of rural tourism and points out that brand competitiveness is the ability of brands to better meet the needs of consumers than competitors in the market competition and create more value advantages for enterprises in a certain market environment. Brand competitiveness mainly reflects the value advantages that brands bring to enterprises and customers. Brand value is not only the cause dimension of brand competitiveness but also the result dimension of brand competitiveness. Therefore, the quantitative research on brand competitiveness and brand value are very similar in many aspects, such as factor selection, method establishment, model setting, etc., which makes the quantification of brand competitiveness concrete and feasible.

The BP neural network model used in this study is best at making decisions in the approximate, uncertain, and even contradictory knowledge environment. It is very suitable for the evaluation and prediction of multiple index system, and can solve the artificial weight design and the calculation of correlation coefficient. BP neural network model is a good method to solve the multiple index rural tourism brand competitiveness evaluation model. This article makes a case study on the competitiveness of rural tourism brands to verify the superiority and effectiveness of the model.

The evaluation of brand competitiveness from the perspective of brand value is a relatively new research point of view. This study also has some limitations and defects, which need to be enriched and improved. It is a demonstration method of the relationship between brand value and brand competitiveness of rural tourism. This study is only a theoretical and logical discussion of the relationship between the two, which inevitably leads to the limitation of insufficient reasoning. If we can use a research method to establish the correlation model between rural tourism brand value and brand competitiveness and make an empirical test, the conclusion will be more convincing. The index system of rural tourism brand competitiveness in this study is only a factor in common sense. It has not been further discussed and defined for the specific brand value factors of different industries and enterprises, and needs more in-depth research and demonstration.[6].

## Figures and Tables

**Figure 1:** The technical route of the rural tourism brand value management model under the big data perspective.

**Figure 2:** BP neural network model structure for rural tourism brand competitiveness assessment.

**Figure 3:** Neural network training process.

**Table 1:** Analysis of brand competitiveness evaluation index system.

Target layer		Criteria layer	Factor layer
Brand competitiveness A	The enterprise value advantage of the brand	Brand's market position B1	Market possession ability C1
			Extra profitability C2
			Market stability C3
		Inside the enterprise support advantage B2	Brand quality support C4
			Brand technology innovation C5
			Brand resource financing C6
			Brand marketing power C7
		Brand development advantage B3	Brand strategic investment degree C8
			Brand growth index C9
			Extend new product acceptance C10
		Brand awareness B4	Awareness without prompting C11
			Awareness after prompting C12
			Subjective familiarity C13
		Brand associative B5	Function associative C14
			Organization associative C15
			Brand uniqueness C16
		Brand recognition B6	Brand symbol awareness C17
			Brand image awareness C18
		Customer loyalty B7	Brand price loyalty C19
			Brand behavior loyalty C20
			Brand trust C21
	Brand customer value advantage	Functional value advantage B8	Product attribute satisfaction function C22
			Product performance satisfaction function C23
			Product quality satisfaction function C24
			Product safety satisfaction function C25
		Emotional value advantage B9	Experiential benefits C26
			Symbolic benefits C27
			Consumer satisfaction with heart needs C28
		Monetary value evaluation advantage B10	Perceived price benefit C29

**Table 2:** Learning sample data after dimensionless processing.

	*B*	*G*	*H*	*I*	*A*	*C*	*E*	*D*	*F*
C1	0.6031	0.8223	0.7189	0.6431	0.3923	0.7089	0.5231	0.6523	0.3589
C2	0.6373	0.8673	0.7524	0.6673	0.5173	0.6924	0.6073	0.6773	0.5024
C3	0.5916	0.8516	0.7989	0.7016	0.5616	0.6989	0.6016	0.6716	0.4989
C4	0.7226	0.7626	0.7224	0.6526	0.6326	0.7324	0.7026	0.7526	0.6224
C5	0.4831	0.7623	0.7789	0.7031	0.4623	0.7589	0.4831	0.7023	0.3789
C6	0.5373	0.6773	0.7824	0.6973	0.4573	0.7624	0.4773	0.6973	0.3824
C7	0.6116	0.8916	0.7889	0.6216	0.6116	0.6589	0.4716	0.7016	0.3689
C8	0.6726	0.7626	0.8024	0.7826	0.5126	0.7824	0.7026	0.7426	0.6024
C9	0.5831	0.7823	0.6089	0.6931	0.5423	0.6789	0.4731	0.7023	0.3789
C10	0.4873	0.8173	0.8024	0.4773	0.2673	0.6224	0.3873	0.5873	0.2124
C11	0.4916	0.6516	0.5989	0.5016	0.5116	0.5789	0.4916	0.5216	0.4489
C12	0.6426	0.8426	0.7924	0.6426	0.4926	0.6824	0.5426	0.6626	0.4224
C13	0.6831	0.8923	0.8189	0.6831	0.5223	0.7489	0.6031	0.7223	0.4489
C14	0.5973	0.8173	0.8024	0.6473	0.4973	0.7024	0.5573	0.6973	0.4324
C15	0.6216	0.8116	0.7689	0.6216	0.4716	0.6689	0.5216	0.6416	0.4489
C16	0.5426	0.7526	0.7924	0.7026	0.4026	0.6724	0.4926	0.6626	0.4924
C17	0.5231	0.8023	0.6989	0.5331	0.5023	0.7489	0.5331	0.5223	0.5989
C18	0.5973	0.7473	0.7224	0.6473	0.5973	0.7424	0.6773	0.7273	0.6024
C19	0.5216	0.7016	0.6489	0.5316	0.5116	0.6789	0.5216	0.6616	0.5289
C20	0.4626	0.6526	0.6224	0.5026	0.4226	0.6024	0.5126	0.6226	0.5424
C21	0.6131	0.8623	0.7989	0.6031	0.5023	0.6689	0.5231	0.7023	0.3789
C22	0.5873	0.7873	0.7624	0.5873	0.4373	0.7024	0.4773	0.6873	0.4024
C23	0.5816	0.7816	0.7889	0.5416	0.5516	0.7089	0.6016	0.7216	0.5689
C24	0.5226	0.8226	0.8024	0.8326	0.8326	0.7524	0.6426	0.7626	0.6224
C25	0.6831	0.8023	0.7789	0.6931	0.6723	0.7389	0.7231	0.7523	0.6789
C26	0.7373	0.7473	0.7324	0.6973	0.7173	0.7124	0.6773	0.7073	0.6924
C27	0.5616	0.7816	0.7189	0.6016	0.5216	0.7189	0.7016	0.7716	0.5189
C28	0.7426	0.7426	0.8124	0.7626	0.7226	0.8224	0.7726	0.8526	0.7224
C29	0.6431	0.6323	0.6489	0.6231	0.6523	0.5589	0.6031	0.6223	0.6989
Output layer A	Medium (010)	Strong (100)	Strong (100)	Medium (010)	Weak (001)	Strong (100)	Medium (010)	Strong (100)	Weak (001)

## Data Availability

The dataset can be accessed upon request.
